The article "The Psychosocial Impact of Dental Esthetics in Undergraduates with Borderline Malocclusion" was retracted in 2023. Reasons: signs of a paper mill; suspected computer-generated content; unreliable results or conclusions; concerns about the data.

# The Psychosocial Impact of Dental Esthetics in Undergraduates with Borderline Malocclusion

**DOI:** 10.1155/2022/2399323

**Published:** 2022-03-08

**Authors:** Hong Zheng, Qingjuan Shi, Wulong Du, Feiou Lin

**Affiliations:** ^1^Department of Orthodontics, School and Hospital of Stomatology, Wenzhou Medical University, Wenzhou, China; ^2^School and Hospital of Stomatology, Wenzhou Medical University, Wenzhou, China

## Abstract

**Background:**

The study investigates the existing correlation between self-perceived malocclusion, the psychosocial impact of dental esthetics, and whether this link involves personality traits.

**Methods:**

The 179 questionnaires from 615 undergraduates in Wenzhou were used for analysis after applying the exclusion criteria. The Psychosocial Impact of the Dental Aesthetics Questionnaire (PIDAQ) was administered to evaluate participants' perceptions of the psychosocial impacts of malocclusion. The need for orthodontic treatment was assessed using the Index of Orthodontic Treatment Need (IOTN). The Chinese version of the Eysenck Personality Questionnaire-Short Scale (EPQ-RSC) evaluated participants' personality characteristics. The Kruskal-Wallis test was used to assess differences between the IOTN-Dental Health Component (DHC) and expectations of orthodontic treatment. Linear regression was applied with PADAQ and its subscale scores against possible variables.

**Results:**

The total and subscale PIDAQ scores were positively correlated with neuroticism. Total PIDAQ scores, the DHC, and the Aesthetic Component (AC) were significantly positively correlated with the subjective AC. The DHC was significantly negatively correlated with extroversion.

**Conclusions:**

We confirmed a modest link between the need for orthodontic treatment and the psychosocial impact of dental esthetics.

## 1. Background

With social and economic development in China, dental health and esthetics are receiving attention from an increasing proportion of the population. Malocclusion can severely affect the appearance of the face and can negatively affect psychological, social, and physical well-being [1–3]. Several studies have reported that patients are often motivated to seek orthodontic treatment to improve their appearance and quality of life [4–6]. The orthodontic treatment of malocclusion improves oral health-related quality of patients' lives [7]. However, many patients who need orthodontic treatment refuse clinical treatment, and dental esthetics may regulate adults' decision-making process for seeking orthodontic treatment [6].

The widely used Psychosocial Impact of Dental Aesthetics Questionnaire (PIDAQ) is designed to assess the psychosocial impact of dental esthetics in orthodontic patients [8]. Several studies have proved the validity and reliability of this scale in various countries and languages, including Chinese [8–10]. Research by Ilijazi-Shahiqi et al. showed that the Albanian version of PIDAQ showed good psychometric characteristics and applicability in Kosovo [11]. Studies by Naseri and others have demonstrated that the Persian version of PIDAQ has the best effectiveness, reliability, and responsiveness in assessing the psychosocial impact of malocclusion on young Iranians [12]. Research by Göranson et al. has shown that the Swedish version of PIDAQ offers good effectiveness and excellent reliability, suitable for future research on the influence of malocclusion on oral health-related quality of life (OHRQoL) of adolescents aged 12 to 19 in Sweden [13]. Nevertheless, some mild malocclusion patients experience severe impacts in daily life that are potentially related to esthetic attitudes and individual personality traits [14]. Furthermore, significant associations have been found between oral health-related quality of life, neuroticism, and extraversion in orthodontic patients [15]. Thus, it is necessary to consider the effects of personality and self-perceived malocclusion in evaluations in addition to the PIDAQ. Some researchers found that age, sex, normative treatment needs, income, and education might affect the self-perception of OHRQoL [16–18].

To reduce these possible sources of interference, we examined university students with a moderate need for treatment in the current study. The study was conducted to investigate whether a link exists between self-perceived malocclusion and the psychosocial impact of dental esthetics and whether this link involves personality traits.

## 2. Materials and Methods

### 2.1. Participants

We designed a cross-sectional study approved by the Health Research Ethics Board of Wenzhou Medical University (WYKQ2018005). Each participant received a full explanation and provided written informed consent before participating in the research.

The sample included 615 undergraduates (45.1% male) aged 18–24 (median, 20; interquartile range, 19–21 years) from Wenzhou, China. Exclusion criteria are as follows [5]: (1) had majored in oral science or professional art; (2) craniofacial anomalies, such as a palate or cleft lip; (3) undergoing or had undergone previous orthodontic treatment; and (4) craniofacial syndromes, items missed out, and refusal to undergo dental inspections. A total sample of 179 questionnaires was used for analysis after applying the exclusions described in the methods.

### 2.2. Psychosocial Impact of Dental Aesthetics Questionnaire (PIDAQ)

The PIDAQ was administered to evaluate participants' perceptions of the psychosocial impacts of malocclusion [19]. This questionnaire includes four subscales: Social Impact (SI, eight items), Aesthetic Concern (AC, three items), Dental Self-Confidence (DSC, six items), and Psychological Impact (PI, six items). A five-point Likert scale was applied for rating each item. The response options were defined as follows: 0, not at all; 1, a little; 2, somewhat; 3, strongly, and 4, very strongly. Each subscale score was obtained by summing the item scores. A reversed dental confidence (DC) score was adapted in the present study to find a continuous measure of impact and keep the scores of all questionnaire items in the same direction.

### 2.3. The Chinese Version of the Eysenck Personality Questionnaire-Short Scale (EPQ-RSC)

EPQ-RSC is reported to be more applicable in China than the full version. Therefore, it was used to assess the personality traits of participants in this study [20]. This scale contains 48 questions with yes and no options consisting of four dimensions of temperament, such as extroversion/introversion (E), neuroticism/stability (N), psychoticism/socialization (P), and the Lie scale (L). Extraversion is characterized by sociability, liveliness, and an outgoing temperament; neuroticism is characterized by emotional instability and anxiety; psychoticism is associated with tough-mindedness, aggressiveness, indifference, and egocentricity; and the Lie scale is related to unsophisticated dissimulation and conformity. The raw score of each dimension can be transformed to a *T*-score, where a higher score suggests extroversion, neuroticism, or psychoticism. The corresponding inclinations were defined as follows: ambiversion (43.3–56.7), tendentious type (38.5–43.3 or 56.7–61.5), and typical type (<38.5 or >61.5).

### 2.4. The Index of Orthodontic Treatment Need (IOTN)

The need for orthodontic treatment was assessed according to the IOTN, which consists of the Dental Health Component (DHC) and the Aesthetic Component (AC) [21]. Self-perceived dental esthetics was evaluated by the participants using the IOTN-AC. Participants were presented with a set of 10 colour photographs of the anterior teeth showing varying degrees of malocclusion. They were asked to choose the photograph they felt most closely resembled their dental appearance. Later, the investigators performed oral examinations and used the IOTN-DHC criteria to determine participants' normative treatment needs. Oral examinations were performed by an investigator who had undergone training and calibration (intraexaminer reliability: weighted kappa 0.91). Patients with DHC grade 3, which represented the moderate or borderline need for treatment, were included in the study. Subjective AC grades 1–4 represent no or little need for treatment. Subjective AC grades 5–7 represent a moderate or borderline need for treatment, and subjective AC grades 8–10 illustrate a definite need for orthodontic treatment.

### 2.5. Statistical Analysis

SPSS software (version 22.0; SPSS, Chicago, Ill) was used to analyze research data. A one-way analysis of variance (ANOVA) was performed to evaluate the PIDAQ score using the least significant difference post hoc test. The Kruskal-Wallis test was used to assess differences between IOTN-DHC values and expectations regarding orthodontic treatment. A *t*-test was used to test differences between males and females. *P* < 0.05 was considered significantly different.

## 3. Results

### 3.1. Participants' Demographics

A total sample of 179 questionnaires was used for analysis after applying the exclusion criteria described in the methods. The sample was composed of 74 male and 105 female students, with a mean age of 21.1 ± 1.4 years. The sample included participants with various types of malocclusion (Class I 118, Class II 51, and Class III 10) (Table 1). There were no statistical differences in any variables between males and females (*P* < 0.05), as shown in Table 2.

### 3.2. The Correlation between PIDAQ and Subjective AC as well as Eysenck Personality Inclinations

The total and subscale PIDAQ scores (except dental confidence) were significantly positively correlated with the personality trait of neuroticism. The total PIDAQ scores, AC, and DHC were significantly positively correlated with the subjective AC. The DHC was significantly negatively correlated with the personality trait of extroversion (Table 3).

### 3.3. The Relationship of PADAQ and Its Subscale Scores against Possible Continuous Variables Was Analyzed

The results show a significant difference between extroversion and DHC. Neuroticism was associated with Social Impacts, Psychological Impacts, Aesthetic Concerns, and PADAQ. And the desire for orthodontic teeth of young adults was associated with Social Impacts and DHC. The above indicates that dental esthetics play a vital role in the psychosocial impact of young adults with borderline malocclusion (Table 4).

### 3.4. The Correlation between PIDAQ and the Different Degrees of Neuroticism

Grade 5 *T*-scores indicated significant differences. There were no significant differences between *T*-scores of grades 1, 2, 3, and 4 and PIDAQ (Table 5).

## 4. Discussion

Mckiernan et al. examined adult patients seeking orthodontic therapy and reported a higher proportion of neurotic traits and different attitudes towards malocclusion than the general population [22]. Therefore, elucidating the impact of mental health status and personality tendencies among adult patients should be a routine task for orthodontists. The current study was restricted to college students whose significant life changes were likely to have subsided. Adolescents were omitted because the changes in their primary life can affect the quality of life and make it challenging to identify which daily activities are changed by the need for orthodontic treatment [23].

Most studies have shown no significant difference in the subjective perception of dental attractiveness between men and women. But some previous studies have reported that gender can affect the subjective perception of attractiveness related to teeth and that women are more concerned about their dental appearance, possibly because of the influence of female personality traits [24, 25]. And in our study, there were no differences between male and female college students.

Psychosocial research on the significance of physical attractiveness has suggested a perceived association between beauty and health [26]. The current results revealed that total PIDAQ scores, AC, and DHC were significantly positively correlated with the subjective AC. These findings indicate that college students pay more attention to their teeth because of beauty and health. The findings are consistent with several international studies' results [18, 27] and may be related to increasing media attention to oral science. The current study revealed that different degrees of dental esthetics have different effects on psychology. We found that a grade of 5 exhibited a significant difference compared with the other grades. However, there were no significant differences between grades 1, 2, 3, and 4. This finding indicates that only a certain degree of unsightly dental esthetics will have a psychological impact. Manevska et al. reported that deviation from the normal profile and normal occlusion could affect personal perceptions and emotions, but the range of acceptable facial characteristics is clearly much broader than the norms [28]. This is consistent with the current findings, suggesting that only extreme deformations impact social and psychological factors.

Previous studies have indicated that extraversion and neuroticism are the strongest predictors of subjective well-being, and agreeableness and conscientiousness predispose individuals to a higher level of well-being [29, 30]. Neuroticism involves anger, anxiety, and vulnerability. In one previous study, patients exhibiting neurotic traits were found to have a significantly different perception of their malocclusion compared with a group of adult patients without neurotic characteristics [22]. In addition, it has been reported that individuals who are impulsive, stress-reactive, or socially isolated are more likely to be disappointed with their orthodontic outcomes [32]. Gavric et al. found that self-esteem seems to be influenced by the self-perceived psychosocial impact of dental esthetics in adolescents and young adults [32]. The current study indicated that the more extroverted the character, the lower the need for orthodontic care. And the social and psychological effects of malocclusion deformity in patients with neurotic characteristics were higher than those in other participants.

It should be noted that the results of this study are based on a survey of a sample of college students with relatively similar demographic characteristics. In future studies, we plan to examine people of different ages, professions, and levels of education.

## 5. Conclusion

In summary, we confirmed a modest link between orthodontic treatment needs and the psychosocial impact of dental esthetics. The connection between the psychosocial impact of dental esthetics and the personality trait of neuroticism appeared to be stronger than the link between the psychosocial impact of dental esthetics and the personality trait of extroversion. These findings can provide valuable information for clinical work, making it possible to take measures to minimize adverse effects caused by the patient's psychological state.

## Figures and Tables

**Table 1:** Demographics of the participants.

Demographic	Number	Percentage (%)
Age (y)		
<20	41	22.9
≥20	138	77.1
Gender		
Male	74	41.3
Female	105	58.7
Index of orthodontic treatment		
Moderate (3)	179	100
Malocclusion		
Class I	118	65.9
Class II	51	28.5
Class III	10	5.6
Total	179	100

**Table 2:** Differences between males and females.

	Gender		
	Male	Female	*P* value
PIDAQ	28.5 ± 11.1	30.5 ± 11.8	0.263
SI	4.2 ± 4.7	4.5 ± 5.3	0.638
PI	5.0 ± 3.9	3.9 ± 4.2	0.095
AC	1.6 ± 2.3	1.6 ± 2.4	0.824
DHC	17.8 ± 5.1	18.3 ± 5.3	0.502
Subjective AC	2.3 ± 1.9	2.0 ± 1.2	0.186
TP	47.9 ± 7.9	47.4 ± 8.5	0.678
TE	47.4 ± 10.4	48.6 ± 11.1	0.477
TN	52.3 ± 10.3	50.7 ± 11.2	0.358
TL	48.2 ± 8.7	49.4 ± 9.5	0.411

Abbreviations: PIDAQ: Psychosocial Impact of Dental Aesthetics Questionnaire; SI: Social Impact; PI: Psychological Impact; AC: Aesthetic Concern; DHC: Dental Health Component; TE: *T*-score of extroversion; TN: *T*-score of neuroticism; TP: *T*-score of psychoticism; TL: *T*-score of Lie scale.

**Table 3:** Correlations between variables.

Variable	Subjective AC	TP	TE	TN
PIDAQ total	0.274^∗∗^	0.013	-0.112	0.270^∗∗^
SI	0.104	0.03	0.045	0.255^∗∗^
PI	0.136	-0.017	-0.05	0.243^∗∗^
AC	0.256^∗∗^	0.069	-0.100	0.202^∗∗^
DHC	0.352^∗∗^	0.05	-0.212^∗∗^	-0.024
Subjective AC	1	0.013	-0.13	0.077

Abbreviations: PIDAQ: Psychosocial Impact of Dental Aesthetics Questionnaire; SI: Social Impact; PI: Psychological Impact; AC: Aesthetic Concern; DHC: Dental Health Component; TE: *T*-score of Extroversion; TN: *T*-score of neuroticism; TP: *T*-score of psychoticism. ^∗∗^*P* < 0.01.

**Table 4:** Multivariate regression of PADAQ and its subscale scores against continuous possible variables.

Var	OD		Gender		DS		TP		TN		TE	
Ou	*β* (95% CI)	*P*	*β* (95% CI)	*P*	*β* (95% CI)	*P*	*β* (95% CI)	*P*	*β* (95% CI)	*P*	*β* (95% CI)	*P*
SI	-1.78 (-3.49, 0.08)	0.04^∗^	-0.56 (-2.10, 0.97)	0.47	0.21 (-2.03,2.45)	0.85	0.03 (-0.05, 0.11)	0.51	0.12 (0.06, 0.19)	<0.01^∗∗^	0.05 (-0.01, 0.11)	0.13
PI	-0.76 (-2.20, 0.67)	0.30	-0.46 (-1.74, 0.83)	0.48	0.14 (-1.74, 2.02)	0.89	0.00 (-0.07, 0.08)	0.93	0.11 (.05, 0.16)	<0.01^∗∗^	-0.00 (-0.06, 0.05)	0.88
AC	-0.34 (-1.09, 0.42)	0.38	-0.19 (-0.86, 0.49)	0.59	-0.06 (-1.05, 0.93)	0.91	0.02 (-0.03, 0.06)	0.41	0.06 (0.02, 0.09)	<0.01^∗∗^	-0.02 (-0.05, 0.01)	0.27
DHC	-1.78 (-3.49, -0.08)	0.04^∗^	-0.56 (-2.09, 0.97)	0.47	0.21 (-2.03, 2.45)	0.85	-0.02 (-0.08, 0.12)	0.71	-0.04 (-0.12, 0.03)	0.27	-0.10 (-0.18, -0.03)	<0.01^∗∗^
PIDAQ	-4.06 (-7.78, -0.34)	0.03^∗^	-2.37 (-5.71, 0.97)	0.16	-0.11 (-4.99,4.77)	0.97	0.03 (-0.18, 0.24)	0.78	0.24 (0.08, 0.41)	<0.01^∗∗^	-0.08 (-0.24, 0.08)	0.31

Abbreviations: OD: orthodontic desire; DS: dental student; PIDAQ: Psychosocial Impact of Dental Aesthetics Questionnaire; SI: Social Impact; PI: Psychological Impact; AC: Aesthetic Concern; DHC: Dental Health Component; TE: *T*-score of extroversion; TN: *T*-score of neuroticism; TP: *T*-score of psychoticism. ^∗^*P* < 0.05; ^∗∗^*P* < 0.01.

**Table 5:** Results of one-way ANOVA of factors of Psychosocial Impact of Dental Aesthetics Questionnaire.

*T*-score of N	*n*	Mean ± SD	ANOVA F	LSD post hoc text
Grade 1	24	27.75 ± 10.69	4.22	Grade 5 > 4, 3, 1, 2
Grade 2	23	26.00 ± 8.54		
Grade 3	67	28.37 ± 9.42		
Grade 4	36	29.77 ± 12.53		
Grade 5	29	37.05 ± 14.70		
Total	179	29.67 ± 11.55		

Abbreviations: N: neuroticism; SD: standard deviation; ANOVA: analysis of variance; LSD: least significant difference.

## Data Availability

The data used to support the findings of this study are available from the corresponding author upon request.

## Abbreviations

PIDAQ: Psychosocial Impact of the Dental Aesthetics Questionnaire
SI, eight items: Social Impact
AC, three items: Aesthetic Concern
DSC, six items: Dental Self-Confidence
PI, six items: Psychological Impact
IOTN: Index of Orthodontic Treatment Need
EPQ-RSC: Chinese version of the Eysenck Personality Questionnaire-Short Scale
E: Extroversion/introversion
N: Neuroticism/stability
P: Psychoticism/socialization
L: Lie scale
DHC: Dental Health Component
AC: Aesthetic Component
DC: Dental confidence
ANOVA: One-way analysis of variance.
